# Segmentation of Breast Masses in Mammogram Image Using Multilevel Multiobjective Electromagnetism-Like Optimization Algorithm

This article has been retracted.

**DOI:** 10.1155/2022/8576768

**Published:** 2022-01-17

**Authors:** S. S. Ittannavar, R. H. Havaldar

**Affiliations:** ^1^Department of Electronics and Communication Engineering, Hirasugar Institute of Technology, Nidasoshi, India; ^2^Department of Biomedical Engineering, KLE Dr. MS Sheshgiri College of Engineering and Technology, Belagavi, India

## Abstract

In recent times, breast mass is the most diagnostic sign for early detection of breast cancer, where the precise segmentation of masses is important to reduce the mortality rate. This research proposes a new multiobjective optimization technique for segmenting the breast masses from the mammographic image. The proposed model includes three phases such as image collection, image denoising, and segmentation. Initially, the mammographic images are collected from two benchmark datasets like Digital Database for Screening Mammography (DDSM) and Mammographic Image Analysis Society (MIAS). Next, image normalization and Contrast-Limited Adaptive Histogram Equalization (CLAHE) techniques are employed for enhancing the visual capability and contrast of the mammographic images. After image denoising, electromagnetism-like (EML) optimization technique is used for segmenting the noncancer and cancer portions from the mammogram image. The proposed EML technique includes the advantages like enhanced robustness to hold the image details and adaptive to local context. Lastly, template matching is carried out after segmentation to detect the cancer regions, and then, the effectiveness of the proposed model is analysed in light of Jaccard coefficient, dice coefficient, specificity, sensitivity, and accuracy. Hence, the proposed model averagely achieved 92.3% of sensitivity, 99.21% of specificity, and 98.68% of accuracy on DDSM dataset, and the proposed model averagely achieved 92.11% of sensitivity, 99.45% of specificity, and 98.93% of accuracy on MIAS dataset.

## 1. Introduction

In recent decades, breast cancer is the most common cause of death among women worldwide. The scientific reports show that the early treatment of breast cancer increases the survival rate of the patients [1, 2]. Several imaging modalities are applied for breast cancer detection like X-ray, ultrasound, magnetic resonance imaging (MRI), histology, positron emission tomography (PET), and computerized tomography (CT). [3]. The mammogram image is the best choice among other imaging modalities for breast cancer diagnosis, because of its high reliability and cost-effectiveness. The full-field digital mammography delivers high-resolution high-contrast images, which are useful in improving the performance and efficiency of mammography [4, 5], especially the digital mammographic images are significant in screening the dense breasts, which assist clinicians in the detection of breast cancer types [6]. The manual screening of a mammogram image is costly, tedious, and time-consuming and leads to high false positive rates, due to lack of expertise and variations in tissues [7, 8]. To overcome the aforementioned problems, numerous machine learning algorithms are developed by the researchers, where the techniques include curvelet moments [9], genetic algorithm [10], textural-based mathematical morphology [11], full resolution convolutional network [12], atrous spatial pyramid pooling method [13], generative adversarial network [14], and pixel-wise clustering [15]. However, the existing methodologies are failed to identify the suspicious regions from the mammographic images, due to irregular shapes and appearance of the cancerous cells. The motivation of the research article is to propose a new multiobjective model to overcome the aforementioned problems and to enhance the performance of breast cancer segmentation. The electromagnetism-like (EM) algorithm works mainly based on the stochastic global optimization approach that utilizes mainly the attraction and repulsion mechanism which evaluates the particles optimality. The local search is the most important factor that influences on obtaining accuracy as a solution. The objective function value is determined for one point is by making one point as a worse compared to other particles which are repulsed by them. The total force exerted at each point is evaluated once after the forces of attraction and the repulsion are determined. Based on the EM algorithm, enhancement of the mammographic images is performed for solving the constrained optimization issues.

At first, DDSM and MIAS datasets are used to validate the effectiveness of the proposed model, and then normalization, CLAHE, and median filtering techniques are employed for enhancing the visual ability and contrast of the mammographic images. The median filter is a nonlinear filtering technique that is used to eliminate noise from the images, which helps to improve the performance of segmentation. In the image processing application, the normalization and median filtering techniques are used to preserve the image edges, while removing noise from the images. Correspondingly, the CLAHE significantly improves the brightness of a mammographic image, which helps in better segmentation of noncancerous and cancerous regions. After enhancing the images, segmentation is carried out by using proposed EML algorithm. The proposed multilevel multiobjective EML technique is adaptive to local contexts and robust in preserving the image edge details, when compared to other algorithms, namely, *k*-means, fuzzy *C*-means (FCM) [16, 17], and traditional EML. After segmenting noncancerous and cancerous regions, the segmented image is matched with original ground truth image to analyse the effectiveness of the proposed model by means of Jaccard coefficient, dice coefficient, specificity, sensitivity, and segmentation accuracy. This paper is organized as follows: some papers related to breast cancer detection are reviewed in Section 2. The detailed explanation about the proposed segmentation model and experimental results are given in Sections 3, 4, 5, and 6. The research conclusion is depicted in Section 7.

## 2. Related Works

Bora et al. [18] developed a novel texture gradient-based methodology to segment the pectoral muscle from an image. Initially, the Hough transformation was used to approximate the pectoral edge on probable texture gradient of the mammogram image. Next, polynomial modelling and Euclidean distance regression were used to achieve smooth pectoral muscle curve and the developed method was robust against overlapping and texture fibro glandular tissues. From the experimental investigation, the developed methodology showed better performance in pectoral muscle segmentation by means of accuracy. The developed method failed in the detection of pectoral muscle from the mammogram images, due to lower contrast and smaller size. Shen et al. [19] presented a new model for automatic segmentation of pectoral muscle region from the images. The developed model contains four phases: image preprocessing, genetic algorithm, morphological selection, and polynomial curve fitting. In this literature, genetic algorithm was used to learning multilevel thresholds, and the morphological selection algorithm was used to search the optimal contour of pectoral muscle regions on the basis of morphological features. In this study, mini MIAS, DDSM, and INBreast databases were used to validate the efficiency of the developed model. The detection rate was lower in the developed model, due to dense gland and boundary of the masses.

Zeiser et al. [20] introduced a model on the basis of U-Net to diagnose breast cancer. The developed model contains four phases: image preprocessing, data augmentation, training, and testing. After acquiring the mammogram images from DDSM, image preprocessing was used to enhance the contrast in the images and obtaining region of interest and removing irrelevant information. The data augmentation was used for horizontal mirroring, resizing, and zooming of mammogram images. Lastly, the U-Net method was used for classifying the malignant and benign classes. From the experimental result, it is clear that the developed model achieved better performance in light of dice index, accuracy, sensitivity, and specificity. During detection, U-Net model does not encode the position and orientation of the objects (cancer and noncancer regions) in low-resolution mammogram image. Dong et al. [21] presented a novel automated framework to improve breast cancer detection. Initially, region of interest (ROI) was extracted, and then, rough set method was utilized to enhance the quality of extracted ROIs. Next, the improved vector field convolution features were applied for extracting the feature values from the ROIs. Lastly, random forest classification technique was applied to classify the types of classes, namely, benign and malignant. The major drawback of random forest was its complexity, and also it consumes more time to construct the decision trees.

Sharma et al. [22] developed atlas selection clustering algorithm to identify the variations in mammogram images. The developed algorithm overcomes the problem of poor registration in the mammogram images. The performance of the developed algorithm was validated on two datasets like DDSM and mini MIAS by means of Hausdorff distance and Jaccard index. However, the developed algorithm needs prior information about the images to perform further operations. Rampun et al. [23] developed a pectoral muscle and breast boundary segmentation algorithm for early recognition of breast cancer. At first, the active contour model was applied to detect the breast boundary, and then, postprocessing method was applied to correct the overestimated boundary, which was caused by the artifacts. The canny edge detection technique and a preprocessing methodology were used to detect the pectoral muscle boundary and to eliminate the noisy edges. Next, five edge features were used to search the actual boundary through contour growing. The developed algorithm obtained significant performance by means of dice similarity coefficients compared to manual segmentation. The active contour model failed to segment the nearest objects, due to the interclass distance and larger intraclass variation.

Soulami et al. [24] developed an automated framework for detecting the suspicious portions using the mammographic images. Firstly, two-dimensional median filter was used for enhancing the visual capability of the acquired mammographic images. Further, a novel metaheuristic algorithm named EML was used for segmenting the suspicious portions from the enhanced images. In this literature, MIAS and DDSM datasets were undertaken to validate the effectiveness of the presented model. The major problem in EML algorithm was it consumes more time to the convergence of the parameters like other metaheuristics. Li et al. [25] introduced a novel framework for breast mass segmentation based on U-Net along with attention gates, which contains a decoder and an encoder. The decoder was densely connected with U-Net, which was integrated with attention gates, and the encoder was connected with convolutional network. The developed framework was validated on DDSM database in light of *f*-score, overall accuracy, specificity, and sensitivity. Experimental result shows that the developed framework achieved significant performance in segmentation related to the existing models. The convolutional networks used in the developed model require graphics processing unit system, which was computationally costly. Guo et al. [26] developed a novel approach for mass segmentation in digital mammography on the basis Spiking Cortical Model (SCM) and enhanced Chan and Vese (CV) algorithm. The SCM was applied to achieve mammary specific and to detect the mass edges from the mammogram images. The enhanced CV algorithm combines local region scalable force and physical imaging principle to accurately detect the coarse-to-fine mass boundaries. From the experimental results, the developed approach showed significant performance in mass segmentation compared to the existing approaches in light of specificity, sensitivity, area under the curve, and dice similarity coefficients.

Sathiyabhama et al. [27] developed a novel feature selection framework using a Grey Wolf Optimizer (GWO) for analysing the mammogram image. Thus, to derive the appropriate features from the feature set, the present research work introduces a dimensionality reduction algorithm on the basis of GWO-rough set theory. The dimensionality reduction algorithm will enhance the chosen subsets without the attribute size description automated was not executed.

Shankar and Duraisamy [28] developed a Versatile Duck Traveler Optimization (VDTO) algorithm based on the triple segmentation approaches for performing the segmentation to diagnose the disease. The threshold values are optimized based on the VDTO for multilevel thresholding (MTH) technique for cancer segmentation. The desired region of the breast cancer is determined using VDTO-ROI for tumor region highlighting. However, the developed model needed to extend the VDTO version for disease diagnosing using the medical image processing.

The existing model failed to detect the pectoral muscle, dense gland, and boundary of the masses because of the smaller size and lower contrast of images in low-resolution mammogram image. The active contour model failed to segment the nearest objects, due to the interclass distance and larger intraclass variation. The EML algorithm used in existing researches failed to describe the consumed consumes more time to the convergence of the parameters like other metaheuristics. The dimensionality reduction technique subsets the feature vectors without choosing the attribute size that reduces the detection performance. In the proposed method, the total force exerted at each point, after the forces of attraction and the repulsion are determined. The total force exerted at each point is evaluated once after the forces of attraction and the repulsion are determined. Based on the ELM algorithm, enhancement of the mammographic images is performed for solving the constrained optimization issues. In the segmentation process, the developed method concentrated only on salient regions, where the spurious regions were not considered for segmentation. For overcoming the abovementioned issues and improving the performance of mammographic breast cancer recognition, a new framework is developed in this article.

## 3. Proposed Model

Recently, the breast cancer is a major cancer type among women, where it develops from the breast cells and forms an abnormal mass called as tumor [29]. The tumor cells are majorly divided into two types, benign (partially cancerous) and malignant (cancerous), so early treatment of breast cancer is important in decreasing the fatality rate [30]. The mammographic analysis significantly improves the detection rate and reduces the time consumption compared to other imaging techniques such as PET and CT. The process of finding the suspicious portions from the mammographic images is hard, due to the irregular shapes and appearance of the cancerous cells. In order to highlight this issue and to improve the performance of cancer segmentation, a novel model is developed in this article. Workflow of the proposed model is indicated in Figure 1.

### 3.1. Image Collection

The DDSM and MIAS datasets are used to validate the proposed EML model performance. The DDSM dataset consists of 2620 mammographic images with pixel level ground truth annotation of lesions [31], and the MIAS dataset contains 322 digitalized mammogram images that include abnormal truth marking locations in the images. The MIAS dataset is reduced to 200 micropixel edges, so the size of each mammogram image is 1024 × 1024 [32]. Graphical depiction of DDSM and MIAS databases is denoted in Figures 2 and 3.

### 3.2. Image Denoising

After acquiring the mammogram images, denoising is carried out for enhancing the contrast and visual capability of the mammographic images by using median filter, CLAHE, and normalization techniques. The contrast of the mammographic image is enhanced by varying the pixel values in normalization technique [33]. The mathematical expression of normalization technique is stated in the following equation:

(1) $$\begin{array}{c} \text{Normalization}=\left(I-\mathrm{Min}\right)\times \frac{\text{newMax}-\text{newMin}}{\mathrm{Max}-\mathrm{Min}}+\text{newMin}, \end{array}$$

where original mammographic image is stated as *I*, minimum and maximum pixel value is represented as Min − Max, which ranges from zero to 255. The image normalization technique is a non-linear technique, which operates on the basis of sigmoid function that is represented in the following equation:

(2) $$\begin{array}{c} \text{Normalization}=\left(\text{newMax}-\text{newMin}\right)\frac{1}{1+e^{-\left(I-\beta /\alpha \right)}}+\text{newMin}, \end{array}$$

where *β* is specified as the centered pixel value and *α* is stated as the width of pixel value. Additionally, median filter is applied on the collected mammogram images to remove noise from the images. The median filtering technique is an order statistics filter, which has better noise reduction capability related to other filtering techniques [34]. The median filtering technique replaces the neighbourhood pixel value by the median pixel intensity value in order to eliminate noise from the images. Hence, the median value is calculated using the following equation:

(3) $$\begin{array}{c} \text{median}\left[A\left(x\right)+B\left(x\right)\right]\neq \text{median}\left[A\left(x\right)\right]+\text{median}\left[B\left(x\right)\right], \end{array}$$

where *A*(*x*) and *B*(*x*) are indicated as two different mammogram images. Then, CLAHE is used to improve the brightness of the mammographic images, which helps in the better segmentation of cancerous and noncancerous regions. The CLAHE divides the collected mammogram images into several nonoverlapping blocks, namely, tiles or contextual region, and then, the histogram value is calculated from the contextual regions. Next, the contrast-enhanced intensity histogram and the cumulative probability density of every tile are clipped on the basis of user-defined clip limit. In this study, clip limit is the average number of pixel values falling in each histogram bin and it is the product of the user-defined contrast factor *δ* [35]. The mathematical expression of clip limit is given in the following equation:

(4) $$\begin{array}{c} n_{T}=\left\{\begin{array}{cc} 1, & \frac{\text{if}\delta MN}{L}<1,\\ \frac{\delta MN}{L}, & \text{else}, \end{array}\right.0<\delta \leq 1, \end{array}$$

where *L* is denoted as the number of histogram bins, *M* is indicated as the rows in contextual region, and *N* is stated as the columns in contextual region. The original height of the contextual region histogram *h*_*k*_ is clipped on the basis of *n*_*T*_, as shown in the following equation:

(5) $$\begin{array}{c} h_{k}=\left\{\begin{array}{cc} \;n_{T}, & \text{if }n_{k}\geq n_{T},\\ \;n_{k}, & \text{else}, \end{array}\right.\;k=1,2,\cdots ,L-1, \end{array}$$

where *n*_*k*_ is represented as contextual region histogram. Equation (6) represents the total number of clipped pixels *n*_*c*_.

(6) $$\begin{array}{c} \;n_{c}=MN-\overset{L-1}{\underset{k=0}{\sum }}h_{k}. \end{array}$$

The clipped pixels are distributed back to the histogram bins to renormalize the histogram. In redistribution, the clipped pixels are distributed equally to all the histogram bins, where no bins exceeded clip limit. A number of pixels are selected using Equation (7), which are needed to be distributed to every histogram bin.

(7) $$\begin{array}{c} \;n_{\mu }=\frac{n_{c}}{L}=MN-\frac{\sum_{k=0}^{L-1}h_{k}}{L}. \end{array}$$

At last, Equation (8) represents the renormalized clipped histogram. Graphical depiction of sample-enhanced DDSM and MIAS images is shown in Figures 4 and 5.

(8) $$\begin{array}{c} h_{k}=\left\{\begin{array}{cc} \;n_{T}, & \text{if }n_{k}+n_{\mu }\geq n_{T},\\ \;n_{k}+n_{\mu }, & \text{otherwise}. \end{array}\right. \end{array}$$

### 3.3. Segmentation

After enhancing the mammographic images, the proposed EML algorithm is applied for solving the constrained optimization issues. In this scenario, the proposed EML algorithm is used for segmenting the noncancerous/cancerous portions from the mammographic images, which is mathematically indicated in the following equation:

(9) $$\begin{array}{c} \mathrm{maximize}\;f\left(V\right),V=\left(v_{1},\cdots ,v_{n}\right)\in R^{n},\text{subject to }v\in V, \end{array}$$

where *R*^*n*^ indicates the nonlinear function, *n* indicates the number of pixels, and *V* states the bounded feasible area, which is explained in the following equation:

(10) $$\begin{array}{c} V=\left\{\frac{v\in R^{n}}{l_{i}\leq v_{i}\leq u_{i}},\right.\;i=1,2,\cdots ,n, \end{array}$$

where *l*_*i*_ denotes the lower interval and *u*_*i*_ indicates the upper interval. Hence, *v*_*i*,*g*_ and *N* are applied for exploring *V*, where *g* represents the iteration number which is 100. After the population *S*_*g*_ = {*v*_1,*g*_, ⋯, *v*_*N*,*g*_} is initialized, the EML algorithm runs until the condition for number of iterations is satisfied. The EML algorithm has two steps:

- Step 1: Each point of *s*_*g*_ changes its location using electromagnetism theories of repulsion and attraction
- Step 2: Changed location points are moved locally by using a local search, where it becomes a member of *s*_*g*+1_ members in *g* + 1^th^ generation

Based on electromagnetism theories of repulsion and attraction, the charged particle is defined as *v*_*i*,*g*_ ∈ *s*_*g*_ in the feasible search space *V*. In this scenario, charge of each point is interconnected with cost function, where the cost function is directly proportional to its charge. The points with better cost function are attracted by other points utilizing electromagnetism theories. Lastly, the complete force vectors *F*_*i*_^*g*^are employed to every point along with whole force direction to the location of *y*_*i*,*g*_. The vicinity of every *y*_*i*,*g*_ is explored by exploiting *y*_*i*,*g*_ to *z*_*i*,*g*_ by using a local search. Then, the members *v*_*i*,*g*+1_ of *S*_*g*+1_ of the *g* + 1^th^ generation are achieved using the following equation:

(11) $$\begin{array}{c} v_{i,g+1}=\left\{\begin{array}{cc} y_{i,g}, & \text{if }f\left(y_{i,g}\right)\leq f\left(z_{i,g}\right),\\ z_{i,g}, & \text{otherwise}. \end{array}\right. \end{array}$$

In mammogram segmentation, the thresholding technique is utilized for classifying the grayscale image pixels into distinct sets based on the pixel value *P*. In image segmentation, identifying the optimal threshold is essential, where the selected bilevel thresholding rule of this study is expressed in the following equation:

(12) $$\begin{array}{c} G_{1}⟵p_{i}\text{ if }0\leq p_{i}<\text{th},\\ G_{2}⟵p_{i}\text{ if th}\leq p_{i}<P-1, \end{array}$$

where *p*_*i*_ is specified as the pixel intensity of grayscale image and the two distinct sets are denoted as *G*_1_ and *G*_2_. The bilevel thresholding technique is further extended as shown in the following equation:

(13) $$\begin{array}{c} G_{1}⟵p_{i}\text{ if }0\leq p_{i}<{\text{th}}_{1},\\ G_{2}⟵p_{i}\text{ if }{\text{th}}_{1}\leq p_{i}<{\text{th}}_{2},\\ G_{i}⟵p_{i}\text{ if }{\text{th}}_{i}\leq p_{i}<{\text{th}}_{i+1},\\ G_{n}⟵p_{i}\text{ if }{\text{th}}_{n}\leq p_{i}<P-1, \end{array}$$

where {th_1_, th_2_, ⋯, th_*k*_} is indicated as the distinct thresholds. The threshold th values are chosen to segment the cancer regions correctly in a mammogram image by using multilevel and bilevel thresholding. In this research, OTSU thresholding and Kapur technique are used to find the optimal threshold value. The OTSU thresholding and Kapur technique effectively identify the threshold value with reduced number of iterations that significantly diminish the computational complexity of the system.

- The OTSU thresholding technique iterates all the possible threshold values and also it measures the pixel levels that fall in both background and foreground regions. The OTSU thresholding finds the optimal threshold value, when the sum of background and foreground region achieved minimum value after performing more number of iterations [36]
- Kapur is a nonparametric technique, which is used to determine the optimal threshold value [37]. The Kapur technique works on the basis of probability distribution and entropy of the image histogram. The Kapur technique is aimed at finding the optimal th, which maximizes the overall entropy. The entropy value of the mammogram image measures the separability and compactness. The sample segmented image is graphically shown in Figure 6

At last, template matching is applied between output and ground truth images to validate the effectiveness of the proposed model. In digital image processing, template matching is used to identify small parts from the images, which match to the ground truth image.

In the present research work, the proposed EML algorithm works mainly based on the stochastic global optimization approach that utilizes mainly the attraction and repulsion mechanism which evaluates the particle optimality. The local search is the most important factor that influences on obtaining accuracy as a solution. The objective function value is determined using Equation (13) for one point is by making one point as a worse compared to other particles which are repulsed by them. The total force exerted at each point is evaluated once after the forces of attraction and the repulsion are determined. Based on the ELM algorithm, enhancement of the mammographic images is performed for solving the constrained optimization issues.

## 4. Experimental Result

In this article, the proposed segmentation model performance is simulated by MATLAB (2018a) software tool with Windows 10 operating system (64 bits), 2 TB hard disk, Intel Core i7 processor, and 8 GB RAM. The performance of the proposed model is related with a few benchmark models like U-Net [20], EML [24], and Dense-U-Net with attention gates [25] for evaluating the efficiency of the proposed model over existing models such as FCM, *k*-means clustering, and traditional EML. Additionally, the performance of proposed multilevel multiobjective EML model is analysed in light of Jaccard coefficient, dice coefficient, specificity, sensitivity, and accuracy on DDSM and MIAS databases. Mathematical expressions of Jaccard coefficient, dice coefficient, specificity, sensitivity, and accuracy are denoted in Equations (14), (15), (16), (17), and (18):

(14) $$\begin{array}{c} \text{Jaccard coefficient}\left(\%\right)=\frac{\text{TP}}{\text{FP}+\text{TP}+\text{FN}}\times 100, \end{array}$$

(15) $$\begin{array}{c} \text{Dice coefficient}\left(\%\right)=\frac{2\text{TP}}{2\text{TP}+\text{FP}+\text{FN}}\times 100, \end{array}$$

(16) $$\begin{array}{c} \text{Specificity}\left(\%\right)=\frac{\text{TN}}{\text{FP}+\text{TN}}\times 100, \end{array}$$

(17) $$\begin{array}{c} \text{Sensitivity}\left(\%\right)=\frac{\text{TP}}{\text{FN}+\text{TP}}\times 100, \end{array}$$

(18) $$\begin{array}{c} \text{Accuracy }\left(\%\right)=\frac{\text{TP}+\text{TN}}{\text{TP}+\text{TN}+\text{FP}+\text{FN}}\times 100, \end{array}$$

where  TN, TP, FP, and FN are indicated as the true negative, true positive, false positive, and false negative, respectively.

## 5. Quantitative Performance on DDSM Database

The DDSM database is used to validate the effectiveness of the proposed multilevel multiobjective EML model. In Tables 1 and 2, the effectiveness of the proposed model is validated by means of Jaccard coefficient, dice coefficient, specificity, sensitivity, and segmentation accuracy. In DDSM database, the performance investigation is done for 2620 mammographic images. In Table 1, the effectiveness of proposed multilevel multiobjective EML model is investigated in light of Jaccard coefficient and dice coefficient. In this scenario, the effectiveness of the proposed segmentation model is related with a few existing models such as *k*-means clustering, FCM, EML with OTSU thresholding, and EML with Kapur. Table 1 shows that the proposed model achieved 88.44% of Jaccard coefficient in benign class and 89% of Jaccard coefficient in malignant class, which are better related to the comparative techniques, namely, *k*-means clustering, FCM, EML with OTSU thresholding, and EML with Kapur. Similarly, the proposed multilevel multiobjective EML model achieved 93.87% and 94.18% of dice coefficient in both benign and malignant classes, which are higher related to the comparative techniques. The graphical presentation of the developed multilevel multiobjective EML model by means of Jaccard and dice coefficients on DDSM dataset is represented in Figure 7.

Table 2 shows that the performance of the proposed multilevel multiobjective EML model is analysed in light of specificity, sensitivity, and accuracy. In benign class, the proposed model attained 92.2% of sensitivity, 99.12% of specificity, and 98.65% of accuracy. Correspondingly in malignant class, the proposed model achieved 92.58% of sensitivity, 99.3% of specificity, and 98.72% of accuracy, which are better compared to the existing models *k*-means clustering, FCM, EML with OTSU thresholding, and EML with Kapur. The proposed multilevel multiobjective EML model uses both Kapur and OTSU objective functions to find the approximate Pareto optimal sets, which help in segmenting the exact noncancerous and cancerous portions from the mammographic images. The graphical presentation of the developed EML model in terms of sensitivity, accuracy, and specificity on DDSM database is represented in Figure 8.

## 6. Quantitative Performance on MIAS Database

The MIAS database is applied for validating the effectiveness of the developed EML segmentation model with dissimilar segmentation models such as *k*-means clustering, FCM, EML with OTSU thresholding, and EML with Kapur. Tables 3 and 4 show the performance of the proposed multilevel multiobjective EML model in terms of sensitivity, accuracy, specificity, and Jaccard and dice coefficients. In the MIAS database, the experimental evaluation is done for 322 mammogram images.  Table 3 shows the effectiveness of the proposed multilevel multiobjective EML model, which achieved 90.68% of Jaccard coefficient and 94.74% of dice coefficient in benign class and 89.81% of Jaccard coefficient and 94.63% of dice coefficient in malignant class. Graphical analysis of proposed model by means of Jaccard coefficient and dice coefficient on MIAS dataset is represented in Figure 9.

Table 4 validates the performance of the proposed multilevel multiobjective EML model in terms of specificity, accuracy, and sensitivity on MIAS database. The proposed model attained good performance in segmentation compared to the existing techniques, namely, *k*-means clustering, FCM, EML with OTSU thresholding, and EML with Kapur on MIAS dataset. In this study, the proposed model considers random samples from the feasible search space based on the image histograms. These random samples build the particles in the EML context using objective functions like OTSU and Kapur methodologies. The developed segmentation approach significantly finds the threshold value with reduced number of iterations that completely decreases the computational complexity of the system. The graphical presentation of proposed model in terms of specificity, accuracy, and sensitivity on MIAS database is given in Figure 10.

### 6.1. Comparative Study

Table 5 represents the comparative study of the existing and proposed model. Zeiser et al. [20] developed U-Net to diagnose breast cancer by using mammographic images. After collecting the images from DDSM dataset, data augmentation was applied for horizontal mirroring, resizing, and zooming of mammographic images. At last, U-Net method was used for classifying the malignant and benign classes. In the experimental phase, the presented model attained 92.32% of sensitivity, 80.47% of specificity, and 85.9% of segmentation accuracy. Soulami et al. [24] developed a metaheuristic algorithm (EML) for segmenting the suspicious portions from the collected images. In this study, the mini MIAS and DDSM databases were used to validate the effectiveness of the presented model. Experimental outcome shows that the developed model achieved 85% and 91.07% of accuracy on Mini MIAS and DDSM databases. Li et al. [25] developed U-Net along with attention gates for breast mass segmentation. Experimental result shows that the developed framework obtained better performance in segmentation on DDSM database. Sathiyabhama et al. [27] performed hybridization of GWO and rough set for determining the breast cancer masses using the MIAS dataset which obtained accuracy of 96.4% whereas the developed Versatile Duck Traveler Optimization algorithm by Shankar and Duraisamy [28] obtained accuracy of 93% for the DDSM dataset and 86.7% of accuracy for the MIAS dataset. The models failed to perform dimensionality reduction without choosing the subsets for describing the attribute size which was failed that lowered the accuracy values. The presented model almost achieved 78.38% of accuracy, 77.89% of sensitivity, and 84.69% of specificity in breast mass segmentation. Related to these existing works, the multilevel multiobjective EML model has obtained effective performance in breast cancer segmentation using mammographic images by means of sensitivity, accuracy, and specificity.

## 7. Conclusion

In this paper, a new multilevel multiobjective EML segmentation technique is proposed to segment the breast masses from the mammographic images. The proposed segmentation model effectively segments the breast lesion regions compared to the existing clustering models that help physicians in early treatment of breast cancer. In the experimental phase, the effectiveness of the proposed model is evaluated by means of Jaccard coefficient, dice coefficient, specificity, sensitivity, and accuracy, where the proposed model averagely achieved 92.39% of sensitivity, 99.21% of specificity, and 98.68% of segmentation accuracy on DDSM database. Similarly, the proposed segmentation model averagely achieved 92.11% of sensitivity, 99.45% of specificity, and 98.93% of accuracy on MIAS database and it showed minimum of 7.61% and maximum of 20.3% improvement in accuracy compared to the existing models, namely, U-Net, EML, and Dense-U-Net with attention gates. In the future work, an effective deep learning classification methodology is included in the proposed multilevel multiobjective EML model for classifying the substages of breast cancer.

## Figures and Tables

**Figure 1:** Workflow of the proposed model.

**Figure 2:** DDSM dataset: (a) benign and (b) malignant.

**Figure 3:** MIAS dataset: (a) benign and (b) malignant.

**Figure 4:** Enhanced DDSM dataset image: (a) benign and (b) malignant.

**Figure 5:** Enhanced MIAS dataset image: (a) benign and (b) malignant.

**Figure 6:** (a) Denoised mammographic image, (b) breast mass segmented mammographic image, (c) matched mammographic image, and (d) original ground truth mammographic image.

**Figure 7:** Graphical presentation of the proposed segmentation model by means of Jaccard and dice coefficients on DDSM dataset.

**Figure 8:** Graphical presentation of the developed EML segmentation model in terms of sensitivity, accuracy, and specificity on DDSM database.

**Figure 9:** Graphical presentation of the developed EML segmentation model in terms of Jaccard and dice coefficients on MIAS database.

**Figure 10:** Graphical presentation of the developed EML segmentation model in terms of specificity, sensitivity, and accuracy on MIAS database.

**Table 1:** Performance evaluation in light of Jaccard and dice coefficients on DDSM dataset.

DDSM	Methodology	Jaccard coefficient (%)	Dice coefficient (%)
Benign	*k*-means	77.13	79.34
	FCM	79.15	81.54
	EML OTSU	82.12	86.12
	EML Kapur	67.12	71.23
	Proposed multilevel multiobjective EML model	88.44	93.87

Malignant	*k*-means	82.73	93.56
	FCM	74.92	90.68
	EML OTSU	75.41	85.98
	EML Kapur	69.47	81.99
	Proposed multilevel multiobjective EML model	89	94.18

**Table 2:** Experimental evaluation of proposed and existing models in terms of sensitivity, accuracy, and specificity on DDSM database.

DDSM	Methodology	Sensitivity (%)	Specificity (%)	Accuracy (%)
Benign	*k*-means	81.32	88.15	88.82
	FCM	83.45	89.77	89.13
	EML OTSU	85.54	94.15	94.12
	EML Kapur	75.87	88.97	89.61
	Proposed multilevel multiobjective EML model	92.2	99.12	98.65

Malignant	*k*-means	77.03	87.28	95.99
	FCM	69.98	84.33	95.08
	EML OTSU	76.57	87.26	87.68
	EML Kapur	68.91	82.67	85.34
	Proposed multilevel multiobjective EML model	92.58	99.31	98.72

**Table 3:** Performance evaluation in light of Jaccard and dice coefficients on MIAS dataset.

MIAS	Methodology	Jaccard coefficient (%)	Dice coefficient (%)
Benign	*k*-means	58.55	61
	FCM	68.67	81.8
	EML OTSU	69.72	82.16
	EML Kapur	82.30	88.46
	Proposed multilevel multiobjective EML model	90.68	94.74

Malignant	*k*-means	75.98	77.97
	FCM	77.35	83.85
	EML OTSU	76.50	86.69
	EML Kapur	78.80	88.14
	Proposed multilevel multiobjective EML model	89.81	94.63

**Table 4:** Experimental evaluation of the proposed and existing methods in terms of specificity, sensitivity, and accuracy on MIAS dataset.

MIAS	Methodology	Sensitivity (%)	Specificity (%)	Accuracy (%)
Benign	*k*-means	47.12	62.38	77.90
	FCM	65.73	74.90	86.30
	EML OTSU	69.72	79.56	89.79
	EML Kapur	79.30	89.43	95.86
	Proposed multilevel multiobjective EML model	92.32	99.56	98.96

Malignant	*k*-means	77.37	85.37	78.60
	FCM	70.46	84.32	79.73
	EML OTSU	78.34	85.67	87.93
	EML Kapur	77.62	86.85	88.76
	Proposed multilevel multiobjective EML model		99.34	98.89

**Table 5:** Comparative study of existing and proposed model.

Methodology	Datasets	Sensitivity (%)	Specificity (%)	Accuracy (%)
U-Net [20]	DDSM	92.32	80.47	85.95
EML [24]	DDSM	—	—	91.07
	MIAS	—	—	85
Dense-U-Net with attention gates [25]	DDSM	77.89	84.69	78.38
Hybridization of GWO and rough set [27]	MIAS	—	—	96.4
Versatile Duck Traveler Optimization [28]	DDSM	—	—	93
	MIAS	—	—	86.7
Proposed multilevel multiobjective EML model	DDSM	92.39	99.21	98.68
	MIAS	92.11	99.45	98.93

## Data Availability

The [DDSM dataset: https://wiki.cancerimagingarchive.net/display/Public/CBIS-DDSM, MIAS dataset: https://www.kaggle.com/kmader/mias-mammography] data used to support the findings of this study are included within the article.

## References

[1] Vijayarajeswari R., Parthasarathy P., Vivekanandan S., Basha A. A. (2019). Classification of mammogram for early detection of breast cancer using SVM classifier and Hough transform. *Measurement*.

[2] Muduli D., Dash R., Majhi B. (2020). Automated breast cancer detection in digital mammograms: a moth flame optimization based ELM approach. *Biomedical Signal Processing and Control*.

[3] Sapate S., Talbar S., Mahajan A., Sable N., Desai S., Thakur M. (2020). Breast cancer diagnosis using abnormalities on ipsilateral views of digital mammograms. *Biocybernetics and Biomedical Engineering*.

[4] Hai J., Tan H., Chen J. (2019). Multi-level features combined end-to-end learning for automated pathological grading of breast cancer on digital mammograms. *Computerized Medical Imaging and Graphics*.

[5] Kaur P., Singh G., Kaur P. (2019). Intellectual detection and validation of automated mammogram breast cancer images by multi-class SVM using deep learning classification. *Informatics in Medicine Unlocked*.

[6] Dheeba J., Albert Singh N., Tamil Selvi S. (2014). Computer-aided detection of breast cancer on mammograms: a swarm intelligence optimized wavelet neural network approach. *Journal of Biomedical Informatics*.

[7] Sun W., Zheng B., Lure F. (2014). Prediction of near-term risk of developing breast cancer using computerized features from bilateral mammograms. *Computerized Medical Imaging and Graphics*.

[8] Eltoukhy M. M., Faye I., Samir B. B. (2010). Breast cancer diagnosis in digital mammogram using multiscale curvelet transform. *Computerized Medical Imaging and Graphics*.

[9] Dhahbi S., Barhoumi W., Zagrouba E. (2015). Breast cancer diagnosis in digitized mammograms using curvelet moments. *Computers in Biology and Medicine*.

[10] Pereira D. C., Ramos R. P., Do Nascimento M. Z. (2014). Segmentation and detection of breast cancer in mammograms combining wavelet analysis and genetic algorithm. *Computer Methods and Programs in Biomedicine*.

[11] Mughal B., Muhammad N., Sharif M. (2018). Deviation analysis for texture segmentation of breast lesions in mammographic images. *The European Physical Journal Plus*.

[12] Al-antari M. A., Al-masni M. A., Choi M. T., Han S. M., Kim T. S. (2018). A fully integrated computer-aided diagnosis system for digital X-ray mammograms via deep learning detection, segmentation, and classification. *International Journal of Medical Informatics*.

[13] Wang R., Ma Y., Sun W. (2019). Multi-level nested pyramid network for mass segmentation in mammograms. *Neurocomputing*.

[14] Singh V. K., Rashwan H. A., Romani S. (2020). Breast tumor segmentation and shape classification in mammograms using generative adversarial and convolutional neural network. *Expert Systems with Applications*.

[15] Shi P., Zhong J., Rampun A., Wang H. (2018). A hierarchical pipeline for breast boundary segmentation and calcification detection in mammograms. *Computers in Biology and Medicine*.

[16] Punithavathi V., Devakumari D. (2021). A new proposal for the segmentation of breast lesion in mammogram images using optimized kernel fuzzy clustering algorithm. *Materials Today: Proceedings*.

[17] Chaira T. (2021). An intuitionistic fuzzy clustering approach for detection of abnormal regions in mammogram images. *Journal of Digital Imaging*.

[18] Bora V. B., Kothari A. G., Keskar A. G. (2016). Robust automatic pectoral muscle segmentation from mammograms using texture gradient and Euclidean distance regression. *Journal of Digital Imaging*.

[19] Shen R., Yan K., Xiao F., Chang J., Jiang C., Zhou K. (2018). Automatic pectoral muscle region segmentation in mammograms using genetic algorithm and morphological selection. *Journal of Digital Imaging*.

[20] Zeiser F. A., da Costa C. A., Zonta T. (2020). Segmentation of masses on mammograms using data augmentation and deep learning. *Journal of Digital Imaging*.

[21] Dong M., Lu X., Ma Y., Guo Y., Ma Y., Wang K. (2015). An efficient approach for automated mass segmentation and classification in mammograms. *Journal of Digital Imaging*.

[22] Sharma M. K., Jas M., Karale V., Sadhu A., Mukhopadhyay S. (2019). Mammogram segmentation using multi-atlas deformable registration. *Computers in Biology and Medicine*.

[23] Rampun A., Morrow P. J., Scotney B. W., Winder J. (2017). Fully automated breast boundary and pectoral muscle segmentation in mammograms. *Artificial Intelligence in Medicine*.

[24] Soulami K. B., Saidi M. N., Honnit B., Anibou C., Tamtaoui A. (2019). Detection of breast abnormalities in digital mammograms using the electromagnetism-like algorithm. *Multimedia Tools and Applications*.

[25] Li S., Dong M., Du G., Mu X. (2019). Attention Dense-U-Net for automatic breast mass segmentation in digital mammogram. *IEEE Access*.

[26] Guo Y. N., Gao X., Yang Z. (2018). SCM-motivated enhanced CV model for mass segmentation from coarse-to-fine in digital mammography. *Multimedia Tools and Applications*.

[27] Sathiyabhama B., Kumar S. U., Jayanthi J. (2021). A novel feature selection framework based on grey wolf optimizer for mammogram image analysis. *Neural Computing and Applications*.

[28] Shankar R., Duraisamy S. (2021). *Versatile Duck Traveler Optimization (VDTO) Algorithm Using Triple Segmentation Methods for Mammogram Image Segmentation to Improving Accuracy*.

[29] Anuradha P. V., Jose B. R., Mathew J. (2015). Improved segmentation of suspicious regions of masses in mammograms by watershed transform. *Procedia Computer Science*.

[30] Ramani R., Vanitha N. S., Valarmathy S. (2013). The pre-processing techniques for breast cancer detection in mammography images. *International Journal of Image, Graphics and Signal Processing*.

[31] Heath M., Bowyer K., Kopans D. (1998). Current Status of the Digital Database for Screening Mammography. *Digital Mammography*.

[32] Melloul M., Joskowicz L. (2002). Segmentation of microcalcification in X-ray mammograms using entropy thresholding. *CARS 2002 Computer Assisted Radiology and Surgery*.

[33] Koo K. M., Cha E. Y. (2017). Image recognition performance enhancements using image normalization. *Human-centric Computing and Information Sciences*.

[34] Erkan U., Gökrem L., Enginoğlu S. (2018). Different applied median filter in salt and pepper noise. *Computers & Electrical Engineering*.

[35] Joseph J., Sivaraman J., Periyasamy R., Simi V. R. (2017). An objective method to identify optimum clip-limit and histogram specification of contrast limited adaptive histogram equalization for MR images. *Biocybernetics and Biomedical Engineering*.

[36] Yang X., Shen X., Long J., Chen H. (2012). An improved median-based Otsu image thresholding algorithm. *Aasri Procedia*.

[37] Cuevas E., Zaldívar D., Perez-Cisneros M. (2016). Otsu and Kapur Segmentation Based on Harmony Search Optimization. *Applications of Evolutionary Computation in Image Processing and Pattern Recognition*.

